# Certificateless Hybrid Signcryption by a Novel Protocol Applied to Internet of Things

**DOI:** 10.1155/2022/3687332

**Published:** 2022-02-26

**Authors:** Wenzhan Zhang, Yanhui Zhang, Chong Guo, Qi An, Yuming Guo, Ximing Liu, Shijun Zhang, Junjia Huang

**Affiliations:** ^1^University of Science and Technology of China, Hefei 230026, China; ^2^Beijing Chuangan BDsecurity Technology Co., Ltd., Beijing 100160, China; ^3^Internat of Things Security and Trusted Technology Co., Ltd., Xiamen 361106, China

## Abstract

The rapid development of the Internet of Things (IoT) has accelerated the integration of science and technology with life, enabling the public to start enjoying the convenience brought by intelligent living. However, there are multiple resource-constrained sensing devices in IoT, which are always facing various external or internal attacks, making it difficult to ensure the secure transmission of sensitive data in IoT. Therefore, to address the problem of data transmission in resource-constrained devices in IoT, we propose a new certificateless hybrid signcryption scheme for IoT. It is a novel scheme that satisfies confidentiality and unforgeability, showing higher computational efficiency and lower overhead of transmission. To prove that it satisfies the efficent transmission of IoT, we conduct simulation experiments, and the experimental results show that our proposed scheme has higher efficiency than the existing schemes.

## 1. Introduction

The rapid development of IoT has accelerated the integration of science and technology with life, enabling the public to start enjoying the convenience brought by intelligent life. For example, digitalization brought by the smart city has solved the problem of “people” having difficulty in doing their work, and the automation brought by the smart home has reduced the public's household work. The convenience brought by IoT is far more than that. Based on the convenience brought by the Internet of Things, the scale of IoT devices is also a gradually expanding trend. It is applied in all walks of life, and the security of IoT devices is gradually coming to the fore.

A large number of legacy devices are undergoing digital transformation; however, few of them are equipped with the appropriate protection capabilities, making the overall security of the IoT less reliable. As a result, cloud-only protection for the IoT is far from adequate for its security. As the variety of IoT devices grows, providing attackers with a wider range of attack entry points, IoT will face even greater risk challenges, and the importance of its security protection cannot be ignored even more. IoT terminal, because of performance and cost limitations, hardware, and software security protection, cannot be integrated so that it is fully exposed to the network. Active protection is difficult to achieve because of energy-saving and other requirements of the limitations, and it cannot be reported immediately to complete the operational status of end-to-end protection and monitoring, making it vulnerable to attacks. There is a phenomenon that a large number of IoT terminals are “working with illness.” In addressing IoT security, security protection can be provided from the perception layer, transmission layer, and application layer.

The perception layer has various types of devices, which are secured mainly by encryption and authentication to prevent attackers from illegally accessing tags and nodes. Transport layer protection uses strict authentication mechanisms between nodes and security protocols that are closely related to keys. Application layer security protection focuses on securing database access control techniques. Among the many security risks of IoT, the great security risk is the leakage of users' privacy. Hence, when considering protection, the user's privacy is first secured. The current solution is mainly through encryption, signature, and authorization authentication.

Providing information security services is achieved through cryptosystems in cryptography, where cryptosystems ensure the secure transmission of messages between the communicating parties in an untrustworthy environment. Confidentiality and authentication are important parts of cryptosystems to provide information security services. Confidentiality refers to the mapping of readable plaintext transformations to unreadable ciphertext using encryption. Authentication prevents the communicator from denying previous actions by signing and verifying the identity information of the signer. With the rapid development of network information, the previous encryption technology cannot meet the security needs of IoT, for example, when the ciphertext is tampered with during transmission, the receiver still cannot receive the correct message even after decrypting it using the correct key. Of course, the authentication of the sender is also important during the transmission of the message. Hence, the use of encryption or signature alone is not enough to meet the current needs of IoT security, and a combination of signature and encryption is needed.

The traditional method of providing encryption and signature is “sign first, encrypt later,” however, the computation and communication costs are the sum of the two, which is inefficient. The signcryption scheme simplifies the encryption and signature scheme, reducing the cost of computation and communication while improving the efficiency of signature and encryption. IoT devices usually have limited computing power and cannot afford complex calculations. Hence, signcryption technology can effectively ensure the secure transmission of data while not requiring high computing power.

The traditional encryption technology is usually based on public key infrastructure (PKI) to realize the encrypted transmission of data, and the public key is stored in the public key's directory by the certificate authority. Because of the huge number of IoT devices, using PKI to manage the public key management and authentication of IoT devices needs to assume huge computing and storage capacity, however, the hardware and software resources of IoT devices are not enough to support the resource consumption of PKI encryption system. To ensure the secure transmission of IoT data, a certificateless hybrid signcryption mechanism is proposed to reduce the storage, issuance, and verification costs of public key certificates. It improves the previous key escrow problem and the management problem of certificates in traditional public key infrastructure. The main idea of certificateless hybrid signcryption is that the device itself calculates its own public key, and the private key is jointly generated by the key generation center and the device itself, without binding the identity of the device to the public key, which changes the previous problem of public key escrow.

However, the certificateless signcryption scheme also brings some new problems. The frequent operation of bilinear pairing will consume a lot of hardware and software resources, and the devices with limited IoT resources are not enough to support the above operation. Also, the current schemes are not sufficient to meet the security requirements of IoT device data transmission. Therefore, this paper proposes a new certificateless hybrid signcryption scheme for IoT, and the contributions of this paper are as follows:

1. We propose a new certificateless hybrid signcryption scheme
2. We prove that our scheme meets confidentiality and unforgeability
3. We have compared the efficiency with other schemes and found that our scheme has higher efficiency

The paper is organized as follows: Section 2 focuses on the current state of research on IoT and the development of a certificateless hybrid signcryption scheme.  Section 3 focuses on the preparatory knowledge, including the basics of cryptographic theory, such as random oracle machine provable security theory, discrete logarithm, bilinear mapping, etc.  Section 4 describes the details of our proposed scheme.  Section 5 describes the security analysis of the certificateless hybrid signatures and proves it.  Section 6 compares other schemes with the scheme proposed in this paper for efficiency analysis, and finally, Section 7 concludes the above certificateless hybrid signcryption scheme.

## 2. Related Work

In 1997, Zheng introduced the concept of the signcryption mechanism. It breaks the traditional way of encryption followed by signature, and it adopts the way of simultaneous encryption and signature. It reduces a large number of calculations, and thus, it greatly improves the efficiency of communication, enabling the secure transmission of data [1]. In 2003, AL-Riyami and Paterson proposed certificateless cryptography, which was proposed to solve the problem of key escrow in ID-PKC. The private key in certificateless cryptography is a combination of the user's own private key and part of the private key generated by KGC. It no longer uses a certificate to bind the identity, thus solving the problem of key escrow. However, the ensuing public key replacement attacks still threaten information security [2].

In the early days, there was no formal security definition for hybrid encryption, which was only on the application requirements. The formal security definition was not formally proposed until 2004 when the formal security definition of KEM-DEM structure based on hybrid encryption was formally proposed by Cramer et al. It uses a combination of secret key encapsulation mechanism and data encapsulation techniques, thus allowing hybrid ciphers to solve the IND-CCA security problem, and hybrid ciphers are also an actual public key cryptosystem [3].

In 2005, Dent proposed the concept of hybrid signcryption cipher, which is a combination of the advantages of symmetric and public key ciphers, i.e., the hybrid signcryption uses the symmetric key to encrypt the plaintext and public key to encrypt the key needed to be used in the management of the information symmetric cipher because the two encryptions are done separately. Hence, they do not interfere with each other and are independent of each other, thus improving the reliability and security of the encryption [4].

The concept of certificateless signcryption was first introduced by Barbosa et al. in 2008. It is a cryptographic technique that provides certificateless encryption and signature, thus triggering a frenzied pursuit of certificateless signcryption in the cryptographic community to the extent that certificateless signcryption became one of the popular research projects in cryptography. However, they gave schemes whose process was too complicated, causing problems, such as it being too complex, inefficient, and difficult to handle security issues. Subsequently, Aranha et al. [5], Wu et al. [6], and Selvi et al. [7] also improved the scheme one after another, however, all of them had more or fewer problems. Aranha et al. did not have a security-proof process, and Wu et al. did not implement the unforgeable nature.

In 2010, Xie et al. [8] proposed signcryption schemes with identity-based and certificateless public key encryption, which requires only two bilinear pairwise operations for its signcryption process. It greatly reduces the computation time. However, its verified dissatisfaction meets the unforgeability. In the same year, Li et al. [9] also proposed a certificateless signcryption scheme, which claimed to be a provably secure scheme requiring only two bilinear pairs of operations, and it was later verified to be insecure. Liu et al. [10] also proposed a certificateless signcryption scheme, which was based on the standard model and required five bilinear pairs of operations, and it was later noted to be insecure.

In 2011, Sun et al. [11] proposed a certificateless signcryption scheme that uses only one bilinear pair operation, which was later also pointed out to have shortcomings. In the same year, Wenhao Liu et al. [12] also proposed a very efficient certificateless signcryption scheme. It was also found to have some insecurity problems. Also, in 2012, Singh [13] proposed a certificateless hybrid signcryption scheme based on identity security authentication.

In 2013, Swapna et al. [14] proposed an elliptic curve-based authentication sign-off scheme in a way that it is a multiagent that can perform multiple sign-off processes simultaneously. In the same year, Li et al. [15] also proposed a certificateless hybrid signicryption scheme, which proved the unforgeability and confidentiality of their scheme. In 2014, Lai [16] proposed a multiparty hybrid signing scheme suitable for use in firewalls and with multiple participants, which is implemented by signcryption and multiparty encryption techniques, and using this scheme can significantly improve computation and transmission efficiency while ensuring confidentiality and nonrepudiation. In 2015, Zhang et al. [17] proposed a certificateless aggregated signcryption scheme, which can guarantee confidentiality and reduce the complexity and overhead of transmission at the same time.

In 2016, Zhou et al. [18] proposed a publicly verifiable certificateless hybrid signcryption scheme that can guarantee the security of transmission despite certain information leakage, in line with the properties of public verifiability, confidentiality, unforgeability, and resistance to information leakage. In 2017, Xu et al. [19] proposed a bilinear pair-based certificateless hybrid signcryption scheme that combines certificateless and hybrid signcryption mechanisms with adaptability, unforgeability, confidentiality, and high-security performance and computational efficiency, and it is more suitable for use when bandwidth receives limitations. In 2019, Yu et al. [20] proposed an improved certificateless hybrid signcryption scheme with an efficient cipher scheme for cover Sun, which eliminates the dross, absorbs the essence, and achieves nonrepudiation, as well as public verification based on the efficiency of the original scheme, which can maintain efficient operation when resisting attacks.

From the analysis of the above research, the research on certificateless hybrid signcryption has never stopped, and the research on certificateless hybrid sigcryption has been gradually improved and perfected. This paper is a novel certificateless hybrid signcryption scheme based on the previous ones, which satisfies confidentiality and unforgeability, showing high computational efficiency and low overhead of transmission.

## 3. Preliminary

### 3.1. Basic Mathematical Concepts

1. Euler function: for the positive integer *n*, Euler function *ϕ*(*n*) is the number of positive integers less than or equal to *n* that are mutually prime with *n*
2. Euler's theorem: if  n, a is a positive integer and  n, a are mutually prime, then *a*^*ϕ*(*n*)^ ≡ 1(mod *n*)
3. The original root: if  n, a are positive integers and n, a are mutually prime, such that *a*^*d*^ ≡ 1(mod *n*) , if *δ*(*n*, *a*) denotes the smallest positive integer *d* that makes the equation hold, at which point if *δ*(*n*, *a*)=*ϕ*(*n*), then we call a as the original root of mod *n*

## 4. The Discrete Logarithm Puzzles

If, for an integer *b* and a prime number *p* of an original root, a unique index *i* can be found such that *b*=*a*^*i*^(*mod* *p*), where 0 ≤ *i* ≤ *p* − 1 holds, then the exponent *i* is called  *b* of *a* as the base of the modulus *p* of the discrete logarithm.

### 4.1. Bilinear Pairs

Let a large prime *q* < 2^*k*^ , where *k* denotes a security parameter. Let *G*_1_ be an additive cyclic group of order *q*, *G*_2_ be a multiplicative cyclic group of order *q*, *P* be the generator of *G*_1_, and $\hat{e}=G_{1}\times G_{1}⟶G_{2}$ be a bilinear map with the following three properties:

1. Bilinear: ∀*a*, *b* ∈ *Z*_*q*_^*∗*^ and $\hat{e}\left(aP,bP\right)=\hat{e}{\left(P,P\right)}^{ab}$
2. Nondegradability: $\hat{e}\left(P,P\right)\neq 1$
3. Computability: ∀*P*, *Q* ∈ *G*_1_, there exists an efficient algorithm to compute $\hat{e}\left(P,Q\right)$

### 4.2. Mathematical Difficulties

1. DLP (discrete logarithm problem) problem: given any *Q* ∈ *G*_1_ , compute *a* ∈ *Z*_*q*_^*∗*^ such that  *Q*=*aP*.
2. CDH (computational Diffie–Hellman) problem: suppose *a*, *b*∈_*R*_*Z*_*q*_^*∗*^, known as *P*, *P*^*a*^, *P*^*b*^. Compute *P*^*ab*^.
3. BDH (bilinear Diffie–Hellman) problem: given any (*aP*, *bP*, *cP*), where *a*, *b*, *c* ∈ *Z*_*q*_^*∗*^, calculate *e*(*P*, *P*)^*abc*^.
4. DBDH (decisional bilinear Diffie–Hellman) problem: For any unknown *a*, *b*, *c* ∈ *Z*_*q*_^*∗*^, known (*P*, *aP*, *bP*, *cP*) ∈ *G*_1_, and *z* ∈ *G*_2_, whether *e*(*P*, *P*)^*abc*^ = *z*is decided. If so, *O*_*DBDH*_ returns 1, otherwise, *O*_*DBDH*_ returns 0.

## 5. The Proposed Scheme

This chapter gives a new certificateless hybrid signcryption scheme for IoT, and below are the 6 main modules of the scheme.

### 5.1. System Initialization

Select the additive cyclic group  *G*_1_ and the multiplicative cyclic group  *G*_2_ , where |*G*_1_|=|*G*_2_|=*q*, P is the generator of  *G*_1_. Meanwhile, KGC selects a bilinear pair e : *G*_1_ × *G*_1_⟶*G*_2_ , randomly choosing *x*_0_ as the master key and computes  *P*_*pub*_=*x*_0_P as the system public key. Three hash functions are selected,  *H*_1_={0,1}^*∗*^⟶*G*_1_, *H*_2_={0,1}^*∗*^ × {0,1}^*∗*^ × *G*_1_ × *G*_1_ × *G*_1_ × *G*_1_⟶*Z*_*q*_^*∗*^, and *H*_3_=*G*_2_ × *G*_1_ × *G*_1_⟶{0,1}^*∗*^.

### 5.2. User Key Generation

The user randomly selects  *x*_*i*_ as the secret value and calculates  *P*_*i*_=*x*_*i*_*P* as the user's public key.

### 5.3. Generation of Partial Private Keys

The user sends itself ID to KGC, which calculates  *Q*_*i*_=*h*_1_(*ID*_*i*_) and *d*_*i*_′=*x*_0_*Q*_*i*_. The private secure channel is then used to send *d*_*i*_′ sent to the user.

### 5.4. Generate All User Private Keys

The user receives the KGC sent  *d*_*i*_′ after calculating a partial private key *D*_*i*_=*x*_*i*_^−1^*d*_*i*_′=*x*_*i*_^−1^*x*_0_*Q*_*i*_. After that, the user combines the secret value generated by itself and the partial private key generated by KGC to generate the complete full private key *SK*_*i*_=(*x*_*i*_, *D*_*i*_).

### 5.5. Signcryption

During the signcryption and signcryption process, it is assumed that the sender's user  *ID* is *ID*_*A*_, the recipient's user  *ID* is  *ID*_*B*_, and the message to be sent is m.

The known sender  *ID*_*A*_ and recipient *ID*_*B*_ have completed the initialization of the key, and they know the system parameters, such as the public key and the system public key of both parties. The specific process is as follows:

1. Randomly choose random values *r* ∈ *Z*_*q*_^*∗*^ , and calculate *R* = *rP*.
2. Calculate  *x* = *e*(*x*_*A*_*Q*_*B*_, *D*_*A*_) , and  y = r*P*_*B*_.
3. Calculate the session key  *k* = *H*_3_(*x*, *y*, *R*), and simultaneously encrypt the data  *m*. Perform symmetric encryption, and compute the ciphertext  *c* = *Enc*(*k*, *m*).
4. Calculate *h* = *H*_2_(*ID*_*A*_, *ID*_*B*_, *P*_*A*_, *P*_*B*_, *P*_*pub*_, *R*).
5. Calculate *s* = *x*_*A*_*h* + *r*. Generate a signed cipher C = (c, R, s) sent to the recipient  *ID*_*B*_.

### 5.6. Unsigncryption

The system public key is the  *P*_*pub*_. The  *ID*_*A*_ is the identity of the sender, and the  *P*_*A*_ is the public key of the sender. Also, the *ID*_*B*_ is the identity of the receiver and *SK*_*B*_ the private key of the receiver. C = (c, R, s) is the ciphertext. The unsigncryption process is as follows:

1. Calculate *x* = *e*(*x*_*B*_*Q*_*A*_, *D*_*B*_) and *y* = *x*_*B*_*R*
2. Calculate the session key  *K* = *H*_2_(*x*, *y*, *R*), simultaneously decrypt the ciphertext c, and calculate the plaintext *m* = *Dec*(*k*, *c*)
3. Calculate *h* = *H*_2_(*ID*_*A*_, *ID*_*B*_, *P*_*A*_, *P*_*B*_, *P*_*pub*_, *R*). Also, verify if the equation *sP* = *hP*_*A*_ + *R* holds

If the validation equation holds, then receive the message *m*. If it does not hold, the message is dropped directly.

## 6. Correctness Analysis

In the scheme of this paper, the correctness analysis is in two parts as follows:

### 6.1. Symmetric Encryption

The first part proves that the session key for symmetric encryption between user A and user B is correct. The parameter *x* calculated by user A is as follows:

(1) $$\begin{array}{c} x=e\left(x_{A}Q_{B},D_{A}\right)=e\left(x_{A}Q_{B},x_{A}^{-1}d_{A}^{\prime }\right)=e\left(Q_{B},d_{A}^{\prime }\right)=e\left(Q_{B},x_{0}Q_{A}\right)=e\left(Q_{A},d_{B}^{\prime }\right)=e\left(x_{B}Q_{A},x_{B}^{-1}d_{B}^{\prime }\right)=e\left(x_{B}Q_{A},D_{B}\right). \end{array}$$

After extrapolation, it can be found to be equal to parameter *x* calculated by user B.

The parameter *y* calculated by user *B* is as follows:

(2) $$\begin{array}{c} y=rP_{B}=rx_{B}P=x_{B}rP=x_{B}R. \end{array}$$

After extrapolation, it can be found to be equal to parameter *y* calculated by user *B,* and *R* is a common parameter known to both user *A* and user *B*. Therefore, the session key computed by user *A* and user *B,K*=*H*_3_(*x*, *y*, *R*), is the same.

### 6.2. Authentication Process

The second part proves that the authentication process of user B to user A's signed secret message is correct. User A and user B calculate the message hash *h* for both *h* = *H*_2_(*ID*_*A*_, *ID*_*B*_, *P*_*A*_, *P*_*B*_, *P*_*pub*_, *R*), where the identity of user A and user B and public keys are known to both parties. The system public key  *P*_*pub*_ is public, and the parameter  *R* is generated by user *A,* however, they are also attached to the ciphertext *c* and passed to user *B*. Therefore, the message hash values computed by user *A* and user B *h* are equal.

User B decides whether to accept the signed message by calculating whether equation *sP*=*hP*_*A*_+*R* or not. If the identity of user A is true, then user A computes the parameter *s* as *s*=*x*_*A*_*h*+*r*, and the authentication equation for user B equals

(3) $$\begin{array}{c} sP=\left(x_{A}h+r\right)P=x_{A}hP+rP=hx_{A}P+rP=hP_{A}+R. \end{array}$$

Verify that the equation holds. Since *x*_*A*_ is the private key of user *A*, only user *A* has it. Then, user *A* alone can compute its public key  *P*_*A*_ corresponding to its public key with the correct parameter *s*. Hence, the correctness of user B's verification equation for user *A* is proven.

## 7. Security Analysis

### 7.1. Confidentiality Analysis

The scheme in this paper establishes a session using a public-private key encryption scheme with KGC, negotiating the session key and transmitting the signature during the session establishment process. The session key is computationally obtained by  *K* = *H*_3_(*x*, *y*, *R*), where *x* = *e*(*x*_*A*_*Q*_*B*_, *D*_*A*_),  *y* = *rP*_*B*_, and *R* = *rP*. The attacker wants to compute to get the session key between user A and user B. He needs to compute to get *x*, *y*, *R*, where *R* is contained in the ciphertext, which is easily intercepted by the attacker. While the attacker does not know the private keys of the two users  *x*_*A*_ and  *x*_*B*_, the computation of *x* is a BDH puzzle. Hence, it is not feasible for the attacker to compute the value of *x*. The attacker needs to know the random number *r* chosen by user A in the process of establishing the session, or the private key of user B to compute *yx*_*B*_, and either computing r by R or  *P*_*B*_ computing  *x*_*B*_, which are discrete logarithmic puzzles and computationally infeasible.

Hence, the attacker is computationally unable to learn the session key between user A and user B, and the communication between them is confidential.

KGC picks the system private key *x*_0_ which is stored only in the KGC and is not transmitted over any channel, and the attacker is able to use it via the system public key  *P*_*pub*_ to compute *x*_0_ for the discrete logarithm puzzle, which is computationally infeasible. Correspondingly, the attacker passes the user's public key *P*_*i*_ to compute the user's private key *x*_*i*_ for the discrete logarithm puzzle, which is also unavailable, and hence, the private keys of the user and KGC are confidential.

### 7.2. Unforgestibility

Unforgestibility means that it is computationally infeasible for other noncluster nodes, masquerading as in-cluster nodes, to generate signature messages that pass verification.

If an attacker wants to forge a valid signcryption ciphertext by masquerading, the secret value  *x*_*i*_ and the random value *r* have to be chosen, and the forged *s* is generated. However, because of the CDH problem, *s* cannot pass the verifying equation *sP*=*hP*_*A*_+*R*, and KGC will not recognize this malicious node. Hence, the attacker cannot send the ciphertext by masquerading as a legitimate node.

If an attacker wants to replace the private key generated by the node, the user key generates the full private key  *SK*_*i*_. The data sources in the process of generating the complete private key are *x*_*i*_ and *d*_*i*_. *d*_*i*_ is transmitted to the user by KGC under a secure channel, and *x*_*i*_ is stored within the user's own node and is not available to the forger. If nongroup members want to forge the identity of user A, they can only do so by capturing the public key  *P*_*i*_, which is transmitted to the user by *P*_*i*_ computing  *x*_*i*_. It is the discrete logarithm puzzle, and there is no effective algorithm for the discrete logarithm puzzle so far. Hence, the scheme in this paper is unforgeable.

### 7.3. Nonrepudiation

Nonrepudiation means that parties in message communication must add information containing their own unique and distinctive information at the time of message transmission data to prevent the denial of the act after the message transmission is completed.

A complete denial resistance mechanism usually consists of two parts: one for the signature part and one for the verification part. The secret key of the signature part is usually the secret key of the sender, which is the sender's own unique and unique information that only the sender of the message holds. It is also the premise and assumption of the denial resistance. The secret key of the verification part is usually the public key of the sender of the message so that the receiver of the message can verify the message.

Encrypting a message with the sender's private key has a four-part effect, which is as follows:

1. Authentication is performed. If receiver B receives a message encrypted with sender A's private key, it can decrypt it with sender A's public key, and if the decryption is successful, receiver B can be sure that the received message is from sender A. It is because if receiver B can decrypt the message with A's public key, it proves that the original message is encrypted with A's private key and only A knows his private key. Thus, sender A encrypts the message with his private key to make his own digital signature.
2. Putting in a fake. An attacker cannot impersonate sender A. If attacker C impersonates A and sends a message, attacker C cannot encrypt the message with A's private key because attacker C does not have sender A's private key, and receiver B cannot decrypt it with sender A's public key. Hence, attacker C cannot impersonate sender A.
3. Denial-proofness so that if a dispute arises between two parties, receiver B can produce the encrypted message and decrypt it with the public key of sender A, thus proving that the message came from A, since it was encrypted with A's secret key, which only A has.
4. Prevent the message from being tampered with. If attacker C intercepts the confidential message during the message transmission, he can decrypt it using A's public key and change the message, however, he cannot achieve his goal. As attacker C does not know A's private key and cannot encrypt the message using A's private key, after attacker C sends the altered message to receiver B, B cannot decrypt the message using A's public key either, and B will not think that the message came from A.

In this design, when user B receives the signed ciphertext *C*=(*c*, *R*, *s*) from user A, he will verify it, where c is the ciphertext *R* is the temporary parameter generated during communication, and *s* is the “digital signature” generated by user A.

The process is as follows:

Firstly, when user A sends a ciphertext by computing *s*=*x*_*A*_*h*+*r*, where  *x*_*A*_ is the private key of user A and *r* is a random value generated at each communication. When user B receives the message sent by user A, verify whether the equation *sP*=*hP*_*A*_+*R* holds, where *P*_*A*_ is the public key of user A held by user B.

It is known that *s*=*x*_*A*_*h*+*r*. Bringing it into the verification equation yields the following:

(4) $$\begin{array}{c} sP=\left(x_{A}h+r\right)P=x_{A}hP+rP=hx_{A}P+rP=hP_{A}+R. \end{array}$$

According to the formula of the user public key *P*_*i*_=*x*_*i*_*P*, it is known that only *x*_*A*_ can make the verification equation hold. As  *x*_*A*_ is the private key of user A, only A knows it, and if a dispute arises between the two parties, user B can take out the encrypted message and decrypt it by user A's public key, thus proving that the message came from A, and user A cannot deny that it sent the signed message, thus achieving the nonrepudiation of the message.

## 8. Efficiency Analysis

Table 1 shows the time complexity of each operation, where *P* denotes the bilinear pair operation, *S* denotes the scalar multiplication operation on an elliptic curve, *A* denotes the addition operation on two elliptic curve points, *E* denotes the exponential operation, and all the above are being calculated and compared as a multiplication product of *M*.

From Table 2, it can be seen that relative to the existing literature, the scheme in this paper does not add a large computational burden to individual signature nodes based on the implementation of group signatures. Thus, the scheme in this paper has good applicability.

The number multiplication operation time on the elliptic curve on a 900KHZ sensor is approximately 2.6s, and considering the latest CortexA9 1.2 GHz microprocessor for smart terminals, the number multiplication operation time on the elliptic curve is approximately 0.00195s. From Table 3, we can see that the calculation time of our scheme is the shortest.

## 9. Conclusion

Numerous IoT devices form a huge network to form the Internet of Things. However, these IoT devices have limited resources and are highly vulnerable to various network attacks. To ensure the secure transmission of sensitive IoT data among IoT devices, we propose a new certificateless hybrid signcryption scheme. From the comparison results, we conclude that the proposed approach offloads the optimized computational structure of the original signature scheme and greatly improves the computational performance. Also, the scheme has high computational efficiency. However, this proposed scheme also uses too much bilinear computation, and the reduced computational stress is not significant enough. This scheme can be investigated again in future work targeting the reduction of the number of bilinear computations.

## Figures and Tables

**Table 1:** Comparison of time complexity of various operations.

Computational	Time complexity
Scalar multiplication operation *S*	1S ≈ 29M
The addition of points *A*	1A ≈ 0.11 M
The bilinear pair operation *P*	1P ≈ 87M
Exponential operation *E*	1E ≈ 21M
Ordinary hashing operation *h*	Neglect

**Table 2:** Comparison of efficiency.

Options	Signcryption			Unsigncryption		
	Dot product operation	Exponential operation	Bilinear operation	Dot product operation	Exponential operation	Bilinear operation
Yu [21]	3	2	2	0	1	6
Jin[22]	3	3	1	3	3	3
Our scheme	3	0	1	3	0	1

**Table 3:** Comparison of time consumption.

Options	Computational complexity	Total time spent (M)	Times (s)
Yu [21]	3M + 3E + 8P	762	0.0512
Jin[22]	6M + 6 E + 4P	480	0.0322
Our solution	6M + 2P	180	0.0121

## Data Availability

No data were used to support this study.
